This article has been retracted.

# Effect and Repair Mechanism of Nano Ag Sponge Dressing Combined with Gelatin-Bletilla Striata Gum/Salvia Miltiorrhiza on Refractory Orthopedic Wounds

**DOI:** 10.1155/2021/8872235

**Published:** 2021-03-30

**Authors:** Chuanjie Jiao, Ming Deng, Yonggang Ma, Geliang Hu

**Affiliations:** ^1^Department of Orthopedics, People's Hospital Yangxin County of Hubei Province, Huangshi 435200, China; ^2^Department of Orthopedics, Renmin Hospital of Wuhan University, Wuhan 430060, China

## Abstract

**Objective:**

To explore the effect and mechanism of the sponge dressing on the healing of refractory orthopedic wound, and the gelatin-Bletilla striata gum/Salvia miltiorrhiza nano Ag (GBS-Ag) sponge dressing was prepared.

**Methods:**

GBS-Ag sponge dressing was prepared by the freeze-drying method. Twenty male SD rats were randomly divided into the control group (Ctrl group) and GBS-Ag group, with 10 rats in each group, and the rats in the two groups were established a model of back wound infection. The Ctrl group was treated with gauze, while the GBS-Ag group was treated with GBS-Ag sponge dressing. Wound healing rate, blood immune indexes, Ag content in each organ, morphological changes of wound, and expression of transforming growth factor-*β*1 (TGF-*β*1) in wound transformation were detected in the two groups of rats.

**Results:**

The mechanical properties of GBS-Ag sponge dressing were all in line with the standard, and it had good killing effect on the conventional strain after being incubated for 24 hours. Compared with the Ctrl group, the healing rate and lymphocyte percentage in the GBS-Ag group were significantly increased on day 4 and day 10 (*P* < 0.05), while the total number of white blood cells and the percentage of neutrophils were significantly decreased (*P* < 0.05). Compared with Ctrl group, the Ag content in liver, spleen, and kidney of rats in the GBS-Ag group was significantly increased (*P* < 0.05). The histological results showed that the Ctrl group lacked collagen fibers in the dermis, and the angiogenesis was not rich, accompanied by a large number of inflammatory cell infiltration. The epidermal repair of rats in the GBS-Ag group was complete and partially keratinized, the dermis was rich in collagen fibers, with elastic fibers and new blood vessels, inflammatory cells were rare, and new hair follicles and thick-walled blood vessels were also observed. The expression of TGF-*β*1 protein in the wounds of rats in the GBS-Ag group was higher than that of the Ctrl group.

**Conclusion:**

GBS-Ag sponge dressing had multiple effects of sterilization and promoting wound healing, and its mechanism may be related to promoting the TGF-*β*1 protein expression.

## 1. Introduction

The healing of refractory wounds caused by large area soft tissue injury in orthopedics is a complex process, which is a dynamic process involving cells, biochemical reactions, and various enzymes, which run through the whole process of skin injury until the wound is completely healed [1]. Wound healing can be divided into four stages: hemostasis, inflammation, proliferation, and regeneration. Under normal functional conditions, these stages occur in an orderly manner and promote wound healing and reduce scarring [2]. One of the factors affecting wound healing is the prevention of infection. When the proliferation of microorganisms in the wound reaches a certain level, it will become infected, which will then cause local inflammatory reaction and signs of systemic infection, leading to general functional decline and secondary injury of the wound, increase the difficulty of wound healing, and even cause systemic diseases. The other factor is the blood supply to the wound tissue, which provides nutrients, inflammatory cells, and oxygen to the wound tissue, which is crucial for wound healing and controlling the proliferation of wound microorganisms [3].

Dressing is produced based on the wetting theory of wound healing, and dressing incubated at the wound site can retain water, which plays an important role in the formation of the connective tissue and granulation tissue. The dressing should have the characteristics of moisturizing, not affecting gas exchange, and acting as a barrier, which should be nontoxic to the body, not causing allergies, easy to be removed, and not sticking to the wound surface [4]. Ag ion has a very good bactericidal function, and 0.005 mg/L trace Ag ion can achieve a certain bactericidal effect and has inhibitory and killing effects on 16 kinds of bacteria including staphylococcus aureus, mold, pneumococcus, E. coli, and candida albicans, with good spectral antibacterial properties [5]. However, if a large amount of Ag ion is ingested, it will cause Ag poisoning. Studies showed that the amount of Ag in the normal human skin is 0.35 mg/kg cell dry weight [6], indicating that low dose of Ag ion is not toxic to humans and animals.

Scientific research found that both gelatin and Bletilla gum had good biocompatibility and degradability. The composite material of these two substances not only has good water absorption, tear strength, and air permeability but also has good histocompatibility [7, 8]. Salvia miltiorrhiza is a kind of traditional Chinese medicine, which has the effects of promoting blood circulation, removing blood stasis, and promoting tissue regeneration. Therefore, the nano Ag sponge dressing combined with gelatin-Bletilla striata gum/Salvia miltiorrhiza (GBS-Ag) was prepared and applied in the healing of orthopedic hard-to-heal wounds in order to explore the healing effect of GBS-Ag sponge dressing on hard-healing wounds.

In this study, nano Ag was utilized to prepare nano Ag sponge dressings, and gelatin-Bletilla striata gum/Salvia miltiorrhiza was compounded into it as a matrix material. GBS-Ag sponge dressing was prepared by the freeze-drying method. The physical and chemical properties and antibacterial properties of GBS-Ag sponge dressing were determined, to explore the effect of GBS-Ag sponge dressing on wound healing in the rat dorsal trauma model and to explore its potential mechanism. It was hoped that this work can provide a scientific basis for the healing of orthopedic hard-to-heal wounds.

## 2. Materials and Methods

### 2.1. Preparation of GBS-Ag Sponge Dressing

- Preparation of sponge matrix solution was as follows. 3% chitosan solution: 3 g chitosan was added to 100 mL 1% glacial acetic acid solution, stirred, mixed, and filtered; 4% polyvinyl alcohol solution: 4 g polyvinyl alcohol was added to 100 mL distilled water, swelled for 30 min, then stirred and mixed in a water bath pot above 50°C, and filtered; chitosan-polyvinyl alcohol mixture was obtained by mixing 3% chitosan solution and 4% polyvinyl alcohol solution at 1 : 1 volume ratio
- Preparation of nano Ag solution was as follows. Silver nitrate solution: 0.5 g Ag nitrate was dissolved in 1 mL distilled water and mixed well. Mixed solution: 1 g glucose, 1 g polyvinylpyrrolidone, 0.2 g sodium hydroxide, and 1 g cetyltrimethylammonium bromide were dissolved in 40 mL distilled water and mixed well. The Ag nitrate solution and the mixed solution were mixed, stirred by magnetic force and placed at 60°C for 2 h. After centrifugated at 30000 rpm for 30 min, Ag nanoparticles were obtained. The particles were dispersed in distilled water and centrifuged again according to the above centrifugation method, repeating 5 times. Finally, the Ag nanoparticles were added to distilled water and prepared into a 600 *μ*g/mL nano Ag solution, which was sealed and stored away from light
- Preparation of GBS compound Chinese medicine solution was as follows. 4 g gelatine and 4 g Bletilla striata gum were, respectively, weighed. 2 mL extracted solution of Salvia miltiorrhiza was weighted. Then, they were dissolved in 100 mL distilled water, heated, stirred, mixed, and cooled
- The GBS-Ag sponge dressing preparation was as follows. 1 mL nano Ag solution was added to 30 mL chitosan-polyvinyl alcohol mixture, stirred by magnetic force; 1 mL glycerin (plasticizer) was added, stirred by magnetic force; 2 mL GBS compound Chinese medicine solution was added, stirred by magnetic force. Then, glutaraldehyde solution (cross-linking agent) was added, stirred by magnetic force. The mixture was poured into the culture dish, and the film was spread. The mixture was frozen at -20°C for 24 h and vacuum freeze-dried for 48 h, and then GBS-Ag sponge dressing was obtained

### 2.2. Determination of Mechanical Properties of GBS-Ag

Porosity measurement: the GBS-Ag sponge dressing was made into a wafer with a diameter of 1 cm, and the thickness was measured with a vernier caliper and weighed as m^1^. The wafer was immersed in absolute ethanol and left for 2 hours to fully absorb the absolute ethanol till saturation, and it was taken out and weighted as m^2^, where *ρ* was the density of ethanol (0.785 g/cm^3^) at 25°C, and *V* was the volume of the wafer before immersion in ethanol. GBS-Ag sponge dressing made into a total of 5 wafer samples for testing, each measurement was repeated 3 times, and the average value was taken.

Measurement of swelling degree: the weight of the wafer-shaped sample was recorded as m^1^, and it was immersed in physiological saline, left for 2 hours to fully absorb the physiological saline till saturation, and it was taken out and weighted as m^2^.

Determination of moisturizing performance: the wafer sample was soaked after the swelling test into a glass drying dish, the weight of the wafer sample was recorded every 1.5 h, and when it was close to the mass before immersed in physiological saline, the time was recorded as moisturizing time (h) of the dressing.

Determination of tensile strength: the GBS-Ag sponge dressing was made into a long strip sample of 50 mm × 15 mm × 1.5 mm, and the tensile strength (MPa) was measured at a crosshead speed (20 mm/min) via a universal tester.

In the above test, a total of 5 samples of GBS-Ag sponge dressing were made for testing, each measurement was repeated 3 times, and the average value was taken.

### 2.3. Determination of Antibacterial Ability of GBS-Ag

The GBS-Ag sponge dressings were made into wafer with a diameter of 1 cm, immersed in 100 mL sterile saline, respectively, placed in an incubator at 37°C, and taken out and dried for 24 h, respectively. The antibacterial activity of GBS-Ag sponge dressing was evaluated with E. coli, pseudomonas aeruginosa, staphylococcus aureus, and candida albicans. The specific steps were as follows: 70 *μ*L bacterial suspension (10^8^CFU/mL) was inoculated on the LB agar plate, and the dried GBS-Ag sponge dressing was applied on the surface of LB agar plate and placed in an incubator at 37°C for 24 h or 48 h. The diameter of the bacteriostatic ring was then measured. A total of 5 samples of GBS-Ag sponge dressing were made for testing, each measurement was repeated for 3 times, and the mean value was taken.

### 2.4. Experimental Animals and Grouping

20 male SD rats aged 8 weeks were purchased from XX Experimental Animal Center, weighing (250 ± 20) g. All rats were fed in an environment of 25°C room temperature, 50% relative humidity, and 12 h/12 h alternating light and dark. After one week of adaptive feeding, all rats were randomly divided into two groups: Ctrl group and GBS-Ag group, with 10 rats in each group. All animal treatment and experimental procedures were in line with the national standards for experimental animals, and this study had been approved by XX Ethics Committee.

### 2.5. Establishment of the Infection Model of Back Wound and Treatment with GBS-Ag Sponge Dressing

The infection model of back wound was established in all rats. The rats were anesthetized by intraperitoneal injection of 50 mg/kg sodium pentobarbital, the prone position was fixed, the back hair was removed, and the rats were disinfected with medical alcohol. A round wound with a diameter of 1 cm, a full-thickness cortex wound was made on the rat's back with a scalpel, and 100 *μ*L of 10^8^ CFU/*μ*L pseudomonas aeruginosa suspension was added to the wound. After 20 min, a 2 cm × 2 cm GBS-Ag sponge dressing was applied to the back wound of rats in the GBS-Ag group, and the bandage was fixed. The wound surface of rats in the Ctrl group was covered with 2 cm × 2 cm medical gauze. The gauze was pretreated by dropping saline and dried, and the bandage was fixed.

### 2.6. Calculation of the Wound Healing Rate and Detection of Blood Immune Indexes

The wound healing condition of rats in each group was photographed on the 4th and 10th day after dressing, and the wound area was measured by ImageJ software.

Tail venous blood was collected on day 0, day 4, and day 10 after dressing and placed in anticoagulant tubes. Percentage of lymphocytes, percentage of neutrophils, and total white blood cells in the blood of rats in each group was determined by automated hematology analyzer.

### 2.7. Histology Detection

Before the rats were sacrificed, the abaxial traumatic site was taken and enlarged by 2 mm, fixed with 4% neutral formaldehyde for 12 h, dehydrated with alcohol at all levels, and transparented with xylene, and the wound tissue was embedded in paraffin. The slicer was used to cut the paraffin block containing tissues into sections of 5 *μ*m, and the slides were used to retrieve and spread the slices for later use.

HE staining: after conventional dewaxing and dehydration, the sections were dyed with hematoxylin for 5 min, washed for 3 times, differentiated with 0.5% hydrochloric alcohol for 7 s, washed for 3 times, dyed with eosin for 1 min, washed for 3 times, dehydrated with various levels of alcohol, and then transparent and sealed with neutral gum.

Masson staining: the sections were treated with xylene and anhydrous ethanol, fixed at 60°C with Bouin's for 1 h and washed for 3 times; Weigert's iron hematoxylin staining was conducted for 10 min, and the sections were washed for 3 times; Biebrich scarlet acid magenta staining was conducted for 15 min, and the sections were washed for 3 times; phosphorous molybdenum pickling was conducted for 15 min, and aniline blue dyeing was conducted for 10 min, and the sections were washed for 3 times; after washed with 1% acetic acid for 5 min, dehydrated with all levels of alcohol, and transparented, the sections were sealed with neutral gum.

Immunohistochemistry: after conventional dewaxing and dehydration, the sections were incubated at room temperature at 3%H_2_O_2_ for 10 min, washed for 3 times, placed in PBS solution, heated to 95°C by microwave for 10 min, and cooled. 5% fetal bovine serum was added to block the sections for 45 min, and TGF-*β*1 primary antibody (1 : 50) was added, incubated at 4°C overnight, washed for 3 times, dropped with secondary antibody, incubated at room temperature for 1 h, and washed for 3 times. After adding SABC complex, the sections were incubated at room temperature for 1 h, washed for 3 times, added with DAB color solution drops, washed away after 10 min, added with hematoxylin for nucleus staining, and 0.5% hydrochloric acid ethanol differentiation was conducted for 7 s, washed for 3 times. After dehydration by different levels of alcohol, transparent and neutral gum sealing were conducted to the sections. Primary antibody, secondary antibody, SABC compound, and DAB chromogenic liquid were purchased from Shanghai Beyotime Company.

The histological features of the wound in each group of rats were observed under Olympus light microscope.

### 2.8. Ag Content Detection

On the 10th day after the dressing, the rats in each group were sacrificed. The livers, kidneys, and spleens were taken, weighed, and added to 10 mL 70% concentrated nitric acid for heating and digestion, after which the volume was determined to 25 mL, and the Ag content was detected by the inductively coupled plasma mass spectrometer, and the equation for calculating the Ag element content was as follows.

Silver content lmg/kgl = (Meter reading)/(Organ weight)(1000%).

### 2.9. Statistical Analysis

All data were expressed as mean plus or minus standard deviation, statistical analysis was performed with SPSS22.0 software, and *t*-test was adopted for comparison between the two groups. *P* < 0.05 indicated that the difference was significant and statistically significant.

## 3. Results

### 3.1. Mechanical Properties and Antibacterial Ability of GBS-Ag

The mechanical properties of the GBS-Ag sponge dressing were determined to be porosity (66.33 ± 4.91) %, swelling degree (13.75 ± 2.13) %, moisture retention time (16.89 ± 1.21) h, and tensile strength (0.19 ± 0.05) MPa.

In Figure 1, when the strain was incubated with the GBS-Ag sponge dressing for 0 h, the diameters of the bacteriostatic rings produced by the incubation of Escherichia coli, Pseudomonas aeruginosa, Staphylococcus aureus, and Candida albicans were (0.6 ± 0.06) mm, (0.4 ± 0.05) mm, (0.3 ± 0.06) mm, and (0.7 ± 0.1) mm, respectively. After 24 hours of incubation, they increased to (12.5 ± 2.7) mm, (11.5 ± 2.6) mm, (10.5 ± 1.3) mm, and (15.9 ± 1.5) mm, respectively. Compared with those at 0 h of incubation, the diameter of the bacteriostatic ring produced by Escherichia coli, Pseudomonas aeruginosa, Staphylococcus aureus, and Candida albicans at 24 h increased considerably (*P* < 0.05). When the strain was incubated with GBS-Ag sponge dressing for 48 h, the diameters of the bacteriostatic rings produced by the incubation of Escherichia coli, Pseudomonas aeruginosa, Staphylococcus aureus, and Candida albicans were (14.9 ± 2.1) mm, (17.9 ± 2.3) mm, (12.8 ± 11.5) mm, and (17.1 ± 2.3) mm, respectively. Compared with those at 24 h of incubation, the diameter of the bacteriostatic rings produced by Pseudomonas aeruginosa when incubated with GBS-Ag sponge dressing for 48 hours significantly increased (*P* < 0.05), with considerable difference. However, there was no considerable difference between the inhibitory ring diameters at 24 h and 48 h produced by Escherichia coli, Staphylococcus aureus, and Candida albicans incubated with GBS-Ag sponge dressing.

### 3.2. Effect of GBS-Ag on Promoting Wound Healing in Rats

When dressing the wound surface of the rats was changed at different time points, it was found that the adhesion between the wound surface and the dressing of the rats in the Ctrl group was relatively close, and it was easy to tear the new skin when the dressing was uncovered. However, the dressings of rats in the GBS-Ag group were not closely connected to the wound surface, which could be easily uncovered without adhesion to the new skin. As shown in Figure 2, scabs of different degrees appeared on the 4th day in both the Ctrl group and the GBS-Ag group, and the wound began to contract, while the wound healing degree of the GBS-Ag group was better than that of the Ctrl group. On the 10th day, the wounds on the back of rats in the GBS-Ag group had basically healed, while those in the Ctrl group had not.

The statistical results of the detection of the abaxial wound healing rate of the two groups were shown in Figure 3. Compared with the Ctrl group, the abaxial wound healing rate of the rats in the GBS-Ag group was significantly increased on the 4th and 10th day (*P* < 0.05), and the differences were statistically significant. The healing rate of the back wound was 0% in both groups on day 0, and the healing rate of rats in the GBS-Ag group was 99.5% on day 10.

### 3.3. Effect of GBS-Ag on the Immune Response

Tail venous blood was collected on day 0, day 4, and day 10 after dressing, and the total number of white blood cells, percentage of neutrophils, and percentage of lymphocytes was measured. As shown in Figure 4, compared with the Ctrl group, the total number of white blood cells and the percentage of neutrophils in the GBS-Ag group were significantly decreased on day 4 and day 10 (*P* < 0.05), while the percentage of lymphocytes was significantly increased (*P* < 0.05), with statistically significant differences. At day 0, there was no significant difference in total white blood cells, neutrophil percentage, and lymphocyte percentage between the two groups.

### 3.4. Effect of GBS-Ag on the Ag Content in Various Organs

The rats were sacrificed on the 10th day after the medicine was applied, and the Ag content in the skin samples, liver, spleen, and kidney tissues of the two groups of rats was detected by mass spectrometry. In Figure 5, the Ag content in the skin, liver, spleen, and kidney tissues of the Ctrl group was 0. The Ag content in the skin, liver, spleen, and kidney tissues of the GBS-Ag group was (0.0089 ± 0.0006) mg/kg, (0.0106 ± 0.0012) mg/kg, (0.0387 ± 0.0014) mg/kg, and (0.0516 ± 0.0030) mg/kg, respectively. Compared with the Ctrl group, the Ag content in the skin, liver, spleen, and kidney tissues of the GBS-Ag group increased significantly (*P* < 0.05), considerable difference, but it was far below the normal range.

### 3.5. Effect of GBS-Ag on Histological Morphology of Rat Wound

HE staining was performed on the back wounds of the two groups of rats. As shown in Figure 6, the epidermis of the injured tissues in the Ctrl group was not repaired, fibrous cells were relatively deficient, blood vessel formation was not abundant, and a large number of inflammatory cells were accompanied by infiltration. The epidermal repair of rats in the GBS-Ag group was complete, and there was partial keratosis, abundant fibroblasts, and a large number of new blood vessels, but very few inflammatory cells, and new hair follicles and thick-walled blood vessels were observed.

Masson staining results of the wounds on the back of rats were shown in Figure 7. The dark blue in the dermal region was collagen fiber, the red was elastic fiber, and the pink was epithelial cell in the epidermal region, which were basically consistent with the results of HE staining. In the Ctrl group, the dermis of the traumatic tissue was deficient in collagen fibers, with a small amount of elastic fibers, and the epithelial cells in the epidermis were not arranged tightly and regularly enough. In the GBS-Ag group, the dermis was rich in collagen fibers and densely arranged, with a large number of elastic fibers, and the epithelial cells in the epidermis were tightly arranged and regular.

### 3.6. Effect of GBS-Ag on the Expression of the TGF-*β*1 Protein in Rat Wounds

In order to explore the mechanism of GBS-Ag dressing promoting wound healing in rats, the expression of the TGF-*β*1 protein in the wound tissues of the two groups of rats was detected by the immunohistochemistry assay. As shown in Figure 8, TGF-*β*1 was mainly distributed in the cytoplasm and on the cell membrane, showing a light brown color. Compared with the Ctrl group, the expression of the TGF-*β*1 protein in the wound tissues of back of rats in the GBS-Ag group was significantly increased, suggesting that the promotion of the wound healing in rats by the GBS-Ag dressing may be related to the increased expression of TGF-*β*1.

## 4. Discussion

Porosity will affect the absorption rate of wound exudate by dressing, and high porosity is conducive to efficient absorption of exudate by dressing from the wound, as well as the transfer and exchange of nutrients and oxygen, which is conducive to wound healing [9]. The porosity of general dressings was about 65%, and that of GBS-Ag in this study was (66.33 ± 4.91) %, higher than that of general dressings. High swelling rate and long moisture retention time mean that the dressing can be locked in moisture. And high tensile strength helps the dressing to incubate on the surface of the wound and does not fall off with body movement. In this study, the swelling degree, moisture retention time, and tensile strength of GBS-Ag sponge dressing were higher than chitosan-aluminum monostearate composite sponge dressing containing asiaticoside prepared by Phaechamud et al. (2015) [10], indicating that GBS-Ag sponge dressing had good mechanical properties. In addition, in this study, the results showed that the lesions incubated with GBS-Ag sponge dressing had better bacteria killing effect on the strains wound healing after 24 h, but the antibacterial ability was not increased more than that at 48 h. The possible reason was that with the increase of time, the low molecular weight chitosan in sponge dressing and the traditional Chinese medicine components degraded slowly. Therefore, it was advisable to change the dressing daily when incubating GBS-Ag sponge dressing.

The rat model of back wound infection was established, the Ctrl group was treated with gauze for wound care, and the GBS-Ag group was treated with GBS-Ag sponge dressing to evaluate the effect of GBS-Ag sponge dressing on wound healing. According to the results of wound healing rate, the wound healing rate of rats in the GBS-Ag group on day 4 and day 10 was significantly higher than that of the Ctrl group, and the wound healing rate of rats in the GBS-Ag group on day 10 was 99.5%. These results showed that GBS-Ag sponge dressing had no toxic and stimulating effects on wound tissue, could prevent infection, kept wound in the moist environment, and effectively promoted wound contraction and healing. According to the blood immune response indexes of the two groups of rats, the total number of white blood cells and the percentage of neutrophils in the GBS-Ag group were significantly lower than those in the Ctrl group on day 4 and day 10, while the percentage of lymphocytes was significantly higher than that in the Ctrl group. It was speculated that the reason might be that GBS-Ag sponge dressing effectively killed pseudomonas aeruginosa and other bacteria on the wound surface and reduced the systemic immune response caused by bacterial infection, which was consistent with the research results of Assadian et al. (2010) [11].

Ag is one of the normal components of human tissues, with usually 0.35 mg/kg dry weight in cells of the skin, 0.4 mg/kg in the kidney, 2.7 mg/kg in the spleen, and 0.7 mg/kg in the kidney [12]. In this study, the Ag content in the skin, liver, spleen, and kidney of rats in the GBS-Ag group was lower than the normal value. After the adoption of GBS-Ag sponge dressing, there was less Ag residue in each organ in the body, which was far below the normal range and would not cause the Ag poisoning to the body. A small amount of residual Ag had bactericidal effect on each organ, which was conducive to the recovery of each organ, and it was similar to the pharmacokinetic results of Ag nanoparticles in rats [13].

During wound healing, angiogenesis significantly promoted wound healing, and nutrients, inflammatory cells, and oxygen were transported to the wound site along with new blood vessels, providing a material basis for wound healing [14]. In this study, the results of HE staining and Masson staining showed that the epidermis of the injured tissues in the Ctrl group was not repaired, the dermis was deficient in collagen fibers, and the formation of blood vessels was not rich, accompanied by a large number of inflammatory cell infiltration, suggesting that the lack of fibrocytes and capillaries led to the inactive repair. The epidermis of rats in the GBS-Ag group was completely repaired, and some keratosis was found, the dermis was rich in collagen fibers, elastic fibers and new blood vessels were abundant, inflammatory cells were rare, and new hair follicles and thick-walled blood vessels were also observed, which suggested that the GBS-Ag group had strong wound repair ability and promoted wound tissue healing and wound angiogenesis, and the low-dose Ag released by GBS-Ag sponge dressings had significant bactericidal effect and reduced wound inflammation. The increase of collagen and elastin also further verified the performance of GBS-Ag sponge dressing in promoting wound repair.

Studies showed that salvia miltiorrhiza could increase the expression of growth factors (such as transforming factor *β*1 and vascular endothelial growth factor), thus promoting the regeneration of the granulation tissue in wounds and positively promoting wound healing [15]. In this study, the expression of the TGF-*β*1 protein in the dorsal wound tissue of rats in the GBS-Ag group was significantly higher than that in the Ctrl group, suggesting that TGF-*β*1 may play an important role in promoting wound repair by GBS-Ag sponge dressing. However, the specific molecular mechanism of TGF-*β*1 remained to be further studied.

## 5. Conclusion

In this study, nano Ag sponge dressing was prepared with nano Ag, and GBS was compounded into the dressing. The sponge dressing prepared by the freeze-drying method with GBS-Ag composite material had multiple functions of sterilization and promoting wound healing, and the mechanism may be related to the promotion of the TGF-*β*1 protein expression. However, there were still some limitations in this study, such as insufficient discussion on molecular mechanism, which would be our main research direction in the future, and it was hoped that this study could provide scientific basis for the healing of refractory orthopedic wounds.

## Figures and Tables

**Figure 1:** The diameter of bacteriostatic ring with GBS-Ag not immersed in saline and immersed in for 24 h and 48 h (^∗^*P* < 0.05, compared with incubation for 0 h; ^#^*P* < 0.05, compared with incubation for 24 h).

**Figure 2:** Wound healing condition of the two groups of rats.

**Figure 3:** Comparison of the wound healing rate between two groups of rats (^∗^*P* < 0.05, compared with the Ctrl group).

**Figure 4:** Comparison of blood immune indexes between two groups of rats. (a) Total number of white blood cells, (a) Percentage of neutrophils. (a) Percentage of lymphocytes (^∗^*P* < 0.05, compared with the Ctrl group).

**Figure 5:** Comparison of the Ag content in various organs of two groups of rats (^∗^*P* < 0.05, compared with the Ctrl group).

**Figure 6:** Comparison of HE staining on the back of the two groups of rats (ruler = 100 *μ*m).

**Figure 7:** Comparison of Masson staining on the back of the two groups of rats. (ruler = 50 *μ*m).

**Figure 8:** Comparison of expression of TGF-*β*1 in the back wounds of two groups of rats via immunohistochemistry (ruler = 100 *μ*m).

## Data Availability

All data, models, and code generated or used during the study appear in the submitted article.
